# Deep Learning Mechanism for Predicting the Axillary Lymph Node Metastasis in Patients with Primary Breast Cancer

This article has been retracted.

**DOI:** 10.1155/2022/8616535

**Published:** 2022-08-10

**Authors:** N. Ashokkumar, S. Meera, P. Anandan, Mantripragada Yaswanth Bhanu Murthy, K. S. Kalaivani, Tahani Awad Alahmadi, Sulaiman Ali Alharbi, S. S. Raghavan, S. Arockia Jayadhas

**Affiliations:** ^1^Department of Electronics and communication Engineering, Sree Vidyanikethan Engineering College, Tirupati, Andra Pradesh 517102, India; ^2^Department of Computer Science and Engineering, Agni College of Technology, Chennai, 600130 Tamil Nadu, India; ^3^Department of Electronics and communication Engineering, Saveetha School of Engineering, SIMATS, Chennai, Tamil Nadu, India; ^4^Department of Electronics and communication Engineering, Vasireddy Venkatadri Institute of Technology, Guntur, Andhra Pradesh 522508, India; ^5^Department of Computer Science and Engineering, Kongu Engineering College, Erode, Tamil Nadu 638060, India; ^6^Department of Pediatrics, College of Medicine and King Khalid University Hospital, King Saud University, Medical City, PO Box-2925, Riyadh 11461, Saudi Arabia; ^7^Department of Botany and Microbiology, College of Science, King Saud University, PO Box-2455, Riyadh 11451, Saudi Arabia; ^8^Department of Botany, University of Texas Health and Science Center at Tyler, Tyler, 75703 TX, USA; ^9^Department of EECE, St. Joseph University, Dar es Salaam, Tanzania

## Abstract

The second largest cause of mortality worldwide is breast cancer, and it mostly occurs in women. Early diagnosis has improved further treatments and reduced the level of mortality. A unique deep learning algorithm is presented for predicting breast cancer in its early stages. This method utilizes numerous layers to retrieve significantly greater amounts of information from the source inputs. It could perform automatic quantitative evaluation of complicated image properties in the medical field and give greater precision and reliability during the diagnosis. The dataset of axillary lymph nodes from the breast cancer patients was collected from Erasmus Medical Center. A total of 1050 images were studied from the 850 patients during the years 2018 to 2021. For the independent test, data samples were collected for 100 images from 95 patients at national cancer institute. The existence of axillary lymph nodes was confirmed by pathologic examination. The feed forward, radial basis function, and Kohonen self-organizing are the artificial neural networks (ANNs) which are used to train 84% of the Erasmus Medical Center dataset and test the remaining 16% of the independent dataset. The proposed model performance was determined in terms of accuracy (Ac), sensitivity (Sn), specificity (Sf), and the outcome of the receiver operating curve (Roc), which was compared to the other four radiologists' mechanism. The result of the study shows that the proposed mechanism achieves 95% sensitivity, 96% specificity, and 98% accuracy, which is higher than the radiologists' models (90% sensitivity, 92% specificity, and 94% accuracy). Deep learning algorithms could accurately predict the clinical negativity of axillary lymph node metastases by utilizing images of initial breast cancer patients. This method provides an earlier diagnostic technique for axillary lymph node metastases in patients with medically negative changes in axillary lymph nodes.

## 1. Introduction

The uncontrolled growth of cells in the breast is called breast cancer. Breast cancer may affect both women and men, although it affects women greater frequency. When compared to other malignancies, breast cancer has been one of the leading causes of mortality among women. Symptoms of breast cancer include changes in the shape and size of the breast, the thickness of the surrounding tissue, crust, scales, and redness of the skin on the breast. Breast cancer is caused by changes in environmental factors, hormones, and lifestyle, which increases the risk factor for breast cancer. Lymphatic fluid from the breast is passed through the lymphatic vessels. If there are cancer cells in the breast, it enters the lymphatic vessels and begins to grow in the lymph nodes. Breast cancer is usually diagnosed after the onset of symptoms, but many people with breast cancer have no symptoms at all. According to the American Cancer Society, by the end of 2021, there will be 291,660 new cases of invasive breast cancer diagnosed and 44,700 deaths occurred. Breast cancer is becoming more common around the world. It is a serious health issue and a source of concern for so many women. Early identification of breast cancer is important for avoiding fatalities. Earlier therapy is needed for the capability to diagnose breast cancer in its initial stages. Early detection necessitates an effective and dependable diagnostic technique that allows clinicians to distinguish benign from malignant breast cancers. The automated detection of breast cancer is significant for the real-world problem in the medical field. Developing an effective and accurate diagnostic approach is essential. Clinical diagnosis is a serious issue in clinical applications. The classifications of breast cancer data can be used to forecast the results of particular diseases and to identify the genetic activity of tumors [1].

Metastasis is the most prevalent cancer-related disease which causes mortality in women with breast cancer, and the most common type of breast cancer metastatic location is the axillary lymph node (ALN) [2]. This ALN metastasis is important for breast cancer patients' medical studies, prognostic assessment, and specific therapy prescription [3]. The occurrence of lymph node metastases is essential for prognosis, pathologic staging, and therapy planning in women with breast cancer [4]. However, various histologic abnormalities, including epithelial hyperplasia, vascular and lymphatic invasion, and necrosis, have been related to an increased risk of lymph node metastasis. Preoperative prognosis of lymph node metastasis might provide useful data for deciding treatments and formulating surgery plans, easing preparatory considerations. For its convenience, comprehensiveness, and harmless nature, preoperative image examination is extremely valuable [5]. The United States plays an important role in identifying breast cancer and determining lymph node metastases [6]. The physical examination did not show the symptoms of the breast cancer, and the radiologists frequently failed to detect metastases in the majority of the patients. However, detection of axillary lymph node metastasis provides a better result for early diagnosis in 20-35% of breast cancer patients [7]. Most of the research study has discovered that a variety of breast cancer features are associated to lymph node metastases. On images, the length between the dermis and the nipple of breast cancer is found to be a critical indicator for lymph node metastasis [8]. This lymph node metastasis is associated to the occurrence of lymphatic invasion and the volume of an initial tumor [9]. Furthermore, higher flexibility of the original tumor as evaluated by elastography was linked to lymph node metastases in breast cancer patients [10].

Breast cancer cells can be identified in the tissues of breast. In the recent year, a plethora of approaches for estimating breast cancer have been discovered. The biopsies are taken from the breast tissues during biopsy screening. The testing produces more reliable outcomes, but this technique for taking the biopsies from the breast is excruciatingly pitiful and painful [11]. As outcomes, most of patients are not interested in this testing. The mammography is the most commonly used tool for estimating breast cancer since it generates 2D projection imaging of the breast. There are two types of mammogram procedures commonly used such as digital mammography and screen-film mammography [12]. Screen-film mammography is used in asymptomatic female breasts. The conventional mammography procedure takes approximately 20 minutes. It is incapable of detecting cancer that is benign. The screening mammography challenge is solved by digital mammography. It is associated with a computing device, as digital mammogram information is stored on a computer. In digital mammography, captured images are processed by image processing techniques to improve the quality of the images. For misdiagnosed samples, digital mammography performs better. Another popular approach, MRI (magnetic resonance imaging), is mostly used for detecting breast cancer [13]. The MRI is a complicated test. It could also miss certain cancers that mammography could have identified. MRI is being used to determine the true dimension of the breast and to detect various diseases in the breast in women who have been diagnosed with breast cancer. It produces great 3D graphics and demonstrates additional functionalities. Deep learning methods, in particular, gained widespread observation for their superior presentation in image recognition duties [14]. Artificially intelligent systems could detect features in clinical images that human specialists rarely notice and could perform quantitative estimates remotely. Because of their benefits in terms of speed, accuracy, and reproducibility, deep learning algorithms are commonly used in image prediction and diagnosis [15]. Predicting lymph node metastases using images of primary tumors and artificial intelligence might have an excellent diagnostic impact. The scope of this research is to explore the possibility of the deep learning models for estimating medically negative axillary lymph node metastases using initial breast cancer images from the input data.

Ultrasound was already routinely utilized to assess the tumor area and identify the ALN level prior to surgery. An analysis revealed that medical T phase and preoperative axillary ultrasound outcomes have been related to ALN condition in patients with newly diagnosed breast cancer, but the diagnostic effectiveness of axillary ultrasound to evaluate ALN condition was poor in such a region [16]. Radiology could automatically extract a huge number of quality image attributes from clinical images that are difficult to recognize with the human eye [17]. Machine learning approaches have been increasingly employed in prediction in the current year, particularly in medical assessment [18]. It enables systems to learn from previous occurrences in order to infer complicated insights from large sets of data. This is an artificial intelligence separator that utilizes a variety of optimal, analytical, and probabilistic methodologies. Generally, this information is well suited to medical applications; mainly those rely on challenges proteome and genomic dimensions. These approaches are most often used to identify and categorize cancers in a wide variety of clinical situations. Machine learning has been employed first and primarily in the diagnosis and treatment of breast cancer [19]. Data mining techniques are a prominent research part of the medical field. It detects and utilizes patterns and interactions across a huge number of factors, as well as forecasts the outcome of a disease based on past instances contained in databases [20]. These techniques are created to estimate the outcomes of diseases, which is the most interesting and challenging task. Massive amounts of healthcare information can be obtained. It is easily available to clinical research organizations because of the utilization of computers driven by automation systems. Information retrieval requires more time when using a typical machine learning approach to harvest information from big datasets. Medical practitioners mainly employ data mining technologies to categorize and explore patterns and connections across a wide range of factors [21].

There have been a number of approaches developed in recent years with the goal of predicting breast cancer in its early stages; however, these approaches do not produce results that are accurate and dependable. In this study, deep learning strategies were suggested as a potential means of providing an accurate prediction of breast cancer in its earlier stages. Methods of evaluation for artificial neural networks include feed forward, radial basis functions, and Kohonen self-organizing algorithms. These methods are used to test artificial neural networks. After then, the outcomes of the prediction are contrasted to the findings of other radiologist approaches. The following strategy for the rest of the paper is as follows: Section 2 presented the related works that have been completed in this field.  Section 3 illustrates the suggested deep leaning mechanism.  Section 4 depicts the results analysis, whereas Section 5 depicts the paper's discussion. Finally, in Section 6, the paper's conclusion is drawn.

## 2. Related Works

Survival of breast cancer prognosis is a challenging task for most researchers. Current research has made great strides in learning related to this field. The study utilized two prominent data mining methods, decision trees and artificial neural networks, as well as a widely used statistical method, the logistic regression model, to construct a predictive model from a massive dataset of more than 200,000 instances. During performance comparison, the study employed 10-fold cross-validation techniques to calculate the unbiased estimation of these three estimation techniques. The results show that the decision tree is the best predictor on the validation dataset, outperforming artificial neural networks by 94.7 percent, logistic regression models by 92.3 percent, and accuracy by 90.3 percent. The comparison of various estimation methods for breast cancer survival utilizing a big database and 10-fold cross-validation gave the predictive power of various data mining methodologies. In the neural network models, the sensitivity analysis has given a better understanding of the relevance of the prognostic variables employed in this research. This method is inaccurate for large datasets and has poor quality for noisy images [22]. K nearest neighbors and support vector machine use a unique method of predicting breast cancer that monitors machine learning algorithms for diagnosing breast cancer through its utilized features. To get an accurate result, the recommended approach uses 10 times cross verification. A compilation of breast cancer diagnostic data from Wisconsin was obtained from the Machine Learning Repository of UCI. The effectiveness of the proposed system is evaluated in terms of the Matthews correlation coefficient, sensitivity, specificity, accuracy, false omission rate, and false discovery rate. Python has become very successful in integrating SVM and categorizing diagnostic data into two categories based on malignancy. At the training stage of SVM, it achieves 99.68% accuracy. The recommended paradigm would be most useful to medical professionals and the general public. The classifier prepared by the supervised machine learning techniques is very useful in the field of clinical diseases and accurate diagnosis [23].

Early recognition usually requires an effective diagnostic procedure, which physicians can use to predict the tumor which is malignant or benign. The study is aimed at evaluating the performance of supervised learning algorithms and their combinations using the voting classification approach. The voting test technique has numerous samples attached for improved classification. The databases were obtained from the University of Wisconsin database. In this study, the classification performance of J48, Nave Bay, and SVM was examined to improve the prognosis model for decision-making systems in breast cancer survival prognosis. To predict breast cancer, the voting classification technique is used, in which all three classification algorithms are combined. The model that combines three different classes would be more reliable and advanced. In total, 235 cases were accurately identified as malignant, while 6 cases were classified incorrectly as benign. The research concluded that integrating all three algorithms by voting technique is the best strategy for diagnosing breast cancer, depending on all trial findings based on accuracy and other characteristics. This method is not suitable for accurate prediction from the large set of dataset [24]. In each cluster, the data sampling is done by using the K-means algorithm, and gene expression values are sampled by PageRank to functional interaction approach. Among the resultant prioritized genes, hub genes were chosen as indicators to determine sample prognosis. Applying the random forest strategy outperforms standard feature extraction methods and uses other network-based predictive gene selection techniques. A functionality analysis revealed that diverse biological activities were concentrated in every cluster, which appears to represent various aspects of tumor growth in a variety of patient categories. Combined together, these findings support the concept of successfully discovering heterogeneous prognostic genes that are complimentary to one another, hence enhancing predictive performance. The suggested methodology for estimating the prognostic of women with breast cancer is superior to Net Rank and coexpression network strategy, as well as classic feature extraction techniques such as Lasso. To prove that grouping heterogeneity samples improves predictive performance. This method can accurately predict functionalities reflecting patient group characteristics. Also, this approach may successfully discover heterogeneity prognosis genes that are complimentary to one another, hence enhancing predictive performance. This method is more complex and does not handle noisy images [25].

Among the 170 women whose receiving first-line tamoxifen therapy for assessable metastasis breast cancer, the immunohistochemical stain (ER) antibody for the estrogen receptor was made using ERID5. The ligand-binding cytosol test was used a few years ago to diagnose ER status. Similar to the volume used for immunohistochemistry, histology in adjacent volumes has always been used to ensure that the tissues used for cytosol testing are adequate and representative of the overall tumor. Six alternative methods were used to measure the amount of staining, and the findings were compared to see which approach yielded the most clinically meaningful results. As indicated by the Lock-Rank analysis, the clinical outcome was evaluated based on both the length of the response to tamoxifen and the type of response determined by the C-square test. The ER immunohistochemistry test outperformed the cytosol test, with all subjective measures of stained evaluation showing statistically important connections with treatment outcomes. The role of progesterone receptor (PR) labeling with antibodies to NCL and PGR was also investigated. The study employed numerous alternative methods of analyzing stained tissue sections in order to determine which one is the most clinically useful. This method is very expensive and the effects of the measurement result are difficult [26]. Data mining is used to identify breast cancer therapy approaches. The software was created to assist oncology doctors in the implementation of therapeutic approaches for women with breast cancer. Ankara Oncology Hospital data from 462 women with breast cancer is utilized to identify therapy options for new patients. This database has been analyzed using the Weka data mining tool. For these datasets, classification techniques are performed one after another, and the outcomes are compared to determine the best medicine used to treat them. The established software application “Therapy Assistance” employs many methods to determine which of these provide the best results for every feature to forecast, as well as Java NetBeans interfaces. In comparison to one another, the hormone therapy result IB1, the radiation and tamoxifen outputs, the chemotherapy output, and the multilayer perceptron demonstrate the greatest prediction accuracy. This study demonstrates that a data mining technique could be a beneficial tool in clinical applications, especially during the therapy decision-making stage [27].

The importance of categorizing cancer sufferers into lower or higher risk clusters has compelled several research groups from bioinformatics and biomedical fields to study and assess the use of machine learning (ML) methodologies. To diagnose breast cancer, both logistic regression techniques and multiclassifiers have been developed. To make deep estimations on breast cancer datasets in a new setting. This research explored the many data mining algorithms that use categorization and may be used for breast cancer information to provide deep estimations. Furthermore, by testing the information on several categories, this work forecasts that the optimization model will deliver great performance. The database of breast cancer, which has received from the machine learning repository of UCI, consists of 570 cases with 32 characteristics. The set of data is initially preprocessed before being given into several categories such as the IBK, simple logistic regression technique, multilayer perceptron, random forest, K-star, decision table, PART, decision trees, REP trees, and multiclass classifiers. The 10-fold validation data is used for training and testing the new models. The acquired results are assessed using several metrics such as accuracy, RMSE error, RMSE error, sensitivity, specificity, ROC curve area, F-measure, and Kappa statistic, and the duration required to develop the system. The study of the findings shows that, of all the classifications, simple logistic regression gives the deep assumptions and generates the right model, providing maximum and precise measurements, followed by some other approaches such as K-star stands for based classifier, IBK is for nearest neighbor classifier, and MLP stands for neural network. Other models yielded lower accuracy when compared to the logistic regression approach. The main purpose of the research is to analyze the comparative performance of multiple data mining approaches for predicting breast cancer diagnosis, therapy, and prognostic and to select the right model. This method is not suitable for exact prediction of the cancer [28].

During diagnosis and prognosis, a customized group classification technique is provided, which is based on the judgments of several classification models, each developed by training patients with comparable molecular features. This technique was applied to three generally accessible breast cancer databases to assess the risk of metastasis in breast cancer individuals. This technique outperforms competing techniques that do not utilize subtype information or utilized only the subtype preset in all three datasets. This technique exhibits high cross-dataset predictive performance, indicating that it will work well in realistic medical settings. This method outperforms existing core group-based classification algorithms in terms of forecast accuracy. Furthermore, the modeling analysis revealed that the individualized group classifications were persistent with the recent understanding subtypes of breast cancer and differentiated metastasis mechanisms that operate on distinct subtypes. As a result of the classification technique presented in this paper, the classification is better structured based on personalized training data, and that classification can be utilized to develop superior prognosis models for advanced diagnosis and treatment. The implementation of this method is difficult and poor efficiency [29].

Breast cancer is most common type of the tumor in which physicians employ medical prognostic indicators to determine therapy choices, and steroids have been utilized for several years. Immunohistochemistry has surpassed all other test methods for evaluating biomarkers. Despite its widespread application, there are still challenges with tissue fixation, interpretation, technique, and measurement. Despite the fact that various indicators have been studied, the estrogen receptors remain the most dependable and clearest examples of a diagnostic predictor. Practically, it is critical that people involved in predicting and interpreting indicators understand the technical problems and are cognizant of how the development of a certain indicator is linked to breast cancer pathology. A false negative or positive result will have an influence on patient care. Following the study of several indicators, ER was a very consistent and excellent example for the prediction of treatment outcomes for breast cancer. HER2 is used as a marker to identify individuals for a particular type of treatment, trastuzumab, but data on responsiveness are limited. Immunohistochemical measurement of these biomarkers may be effective, but the adjustment, technique, and interpretation should be standardized, and the interpreter should be aware of the predicted trends of specific risks and reactions associated with breast cancer pathology. Quantitative PCR is used to measure ER and HER2 gene expression patterns. There are commercialized experiments that address the function of various genes such as Oncotype DX. The application of immunohistochemistry, as well as the measurement challenges associated with it, may undergo significant change if molecular testing were to be automated to the same extent as biochemical tests, and if the cost of the test were comparable to that of competitive tests. In immunohistochemistry, antibodies are used to search a tissue sample for certain antigens, also known as markers. This technique is performed in a laboratory [30].

The clinical characteristics derived from regular blood tests paired with anthropometric measures should be used to detect breast cancer by utilizing diagnostic machine learning algorithms. The roles of different machine learning modules that are selecting features, information division methods, and categorization in determining suitable biological markers for breast cancer detection were investigated; the latest dataset of medical and anthropometric datasets obtained from healthy and cancer patients was analyzed. To establish the importance of different characteristics, several feature extraction and statistically significant analytical approaches are applied. Moreover, by utilizing these characteristics, prominent classifications such as Nave Bayesian, kernel-related support vector machine (SVM), logistic regression, quadratic and linear discriminant, random forest, and K-nearest neighbor (KNN) were constructed and assessed for risk of breast cancer detection. Among the nine characteristics investigated, the outcomes of feature selection procedures show that age, glucose, and resistance are the most useful and relevant markers for breast cancer detection. The KNN classifier achieved higher accuracy (92.2%) compared to the Gaussian SVM technique. This method is not suitable for large-scale database [31]. New biomarkers were determined for breast cancer based on blood testing by analyzing methylation of DNA in a free DNA (cfTNA) cycle from the blood and control of patients with breast cancer. The study examined the stimulatory methylation of seven potential tumor suppressor genes derived from cfDNA (ITIH5, SFRP1, WIF1, SFRP2, DKK3, SFRP5, and RASSF1A). These studies found that ITIH5 and DKK3 stimulant methylation may be utilized as possible biomarkers in diagnostic and verification processes, with 41% sensitivity and 94% and 99% in normal and benign disease controls, respectively. Furthermore, the correlation of such genes with RASSF1A methylation boosted the sensitivities to 67%. According to the findings of this study, the three types of genes (DKK3 with RASSF1A methylation and ITIH5) might be employed as a possible marker in the initial stages of breast cancer prediction. Because it can only forecast the early stages of breast cancer, this approach is not appropriate for the diagnosis of other forms of the disease [32].

Postmodernization is used to evaluate the patient's pathological response prior to neoadjuvant chemotherapy treatment (NAC) by combining tumor hemoglobin characteristics with conventional pathological tumor properties, as evaluated by ultrasound lead Nair-infrared optical tomography (US-NIR). The database of thirty-four patients was divided into 30 training groups (24 tumors) and test groups (12 tumors). Prior to starting treatment, tumor vascularity was examined with US-NIR computation of fully oxidized and deoxidized hemoglobin. Cancer type, Nottingham score, estrogen, progesterone receptors, mitotic index, and human epidermal growing factor receptor 2 features are included in the modeling. They used the Miller-Payne approach to standardize patients' pathological responses. When using only tumor pathological factors for the experimental dataset, their pattern averaged 88.9 percent, sensitivity 56.8 percent, negative prognosis value 70.9 percent, positive prognosis value 84.8 percent ,and recipient side effect curve 84.0 percent. Furthermore, when tHb was added as a prognosticator, the outcomes improved to 80 percent, 95 percent, 91 percent, 87 percent, and 93.5 percent, respectively; then, the oxyHb was added as a component with variance of tumor, and the outcomes were 77 percent, 85 percent, 83 percent, 83 percent, and 90.6 percent, respectively. When compared to employing tumor pathological characteristics only, the findings of this investigation showed that the inclusion of tHb enhanced predicted sensitivity, AUC, and NPV. Furthermore, the model was evaluated on a tiny number of patients, calling the suggested expertise system's dependability into doubt. This strategy is only applied to a small subset of available datasets; if we were to use it with a more extensive collection of data, the predictive accuracy of the model would suffer dramatically [33].

In terms of effectiveness, the ANN model exceeds most prior supervised learning approaches, attaining a 99.57 percentile in the dataset of Wisconsin Breast Cancer. The investigational outcomes using Haberman's Breast Cancer dataset reveal that the suggested strategy is better in terms of precision, achieving 88.24 percent. The outcomes are the highest accuracy those achieved from an artificial neural network in JNN environment with no data preparation. After obtaining the Breast Cancer Wisconsin dataset, the best prediction rate was determined to be 99.57 percent. The values of the parameters were identified, the information was uploaded and divided into training and verifying set, and the appropriate hidden units were determined. The sets were then trained and verified to achieve the highest level of accuracy [34]. Prognosis and chemotherapy benefits were improved by predicting breast cancer criteria by establishing an “intrinsic” model that integrates gene expression. Prognosis was determined using training dataset from 761 patients, and pathologic complete response (pCR) to a taxane plus anthracycline regimen was determined using training dataset from 133 individuals. Using endogenous subtypes and clinical data, a prognostic model for tip-negative breast cancer was developed. The C-index assessments of the joint model performed better than the clinicopathological approach. The intrinsic subgroup method estimates neoadjuvant chemotherapy efficiency with a 97 percent negative predictive value for pCR. In the case of breast cancer, diagnosis by intrinsic subgroup includes valuable predictive and prognostic data to standard measures. In order to make the qRT-PCR test suitable for both prospective and retrospective clinical research, it should be performed on archive breast tissue. The risk of breast cancer cannot be accurately predicted using these methods [35].

The single cell RNA-sequencing, which permits the measurement of transcribed expression patterns in individual cell in a group of cancerous cells, is one major technology which has been used to solve these issues. The researchers looked at scRNASeq cancer classification from a various perspective. This work describes a data analysis method that uses patterns of genetic expression in individual cells to reliably predict six breast cancer cell subtypes. Instead of using the entire human transcript to create diagnostic models, the pipeline first excludes predictions with low exposure and variability. A multivariate regression decreases the number of determinants to 308, of which 34 are longer noncoding RNAs. With nearly 98 percent predictive performance, prediction model optimization reveals that support vector machines and neural networks are the most efficient systems. In general, breast cancer cell type prognosis is related to the patient's survival, so the findings indicate that it has therapeutic value [36]. The study analyzed the ensemble model, such as the combination of random forest, gradient boosting, artificial neural networks, and support vector machines, for breast cancer prediction. For classification, K-means clustering with K-nearest neighbor is used. 1874 patients were tested by using this method, and the accuracy, receiver operating characteristic, and calibration slope were evaluated. The five-year survival rate has been predicted for the patients. The suggested model gives a better result for predicting the survivability of breast cancer [37]. To measure the HER2 overexpression level, the radio immunohistochemical method has been utilized. In the application of this approach, HER2 levels were shown to be higher than normal in 85% of breast cancer tissues. Of those, 23% showed 45 to 480 times higher than normal HER2, which is associated with worsening treatment outcomes. Studies on HER2 levels have produced a number of contradictory effects as a predictor of treatment responsiveness. In general, HER2 hypertension is associated with opposition to hormone treatment, susceptible to resistance to CMF and anthracycline-based chemotherapy. With the introduction of specific anti HER2 drugs, the HER2 level will be significant in providing the most suitable medication regimen for patients. This radiation is very dangerous to the health of the patients [38].

The most important contribution that the research work made can be summarized as follows:

- The dataset of axillary lymph nodes from individuals diagnosed with breast cancer was gathered from the Erasmus Medical Center as well as the national cancer centre
- In order to train and test these datasets, an artificial neural network based on feed forward, radial basis function, and Kohonen self-organizing was utilized
- The values for accuracy, sensitivity, and specificity for the suggested model are figured out. These numbers are then compared to the results of the other four radiologist models. In comparison to other radiologist models, the proposed model attained an accuracy rate of 98 percent

## 3. Methods

### 3.1. Breast Cancer Patient Datasets

The medical records of breast cancer patients were obtained from the Erasmus Medical Center database from February 2018 to July 2021. Totally, 750 cancer patients are selected for the training and validating process with the average age 50 years and ranges between 30 and 75 years. For the internal test, 95 patients are selected with average age of 55 years and range between 32 and 76 years. For the external test, 85 patients are selected with the average age of 50 years and range between 31 and 75 years in Erasmus Medical Center. This research process is illustrated in Figure 1. The clinical information was used to extract initial clinical pathologic data, such as gender, age, pathologic observations, and diagnostic reports. Breast Ultrasonography image datasets at the National Cancer Institute (https://cdas.cancer.gov/datasets/plco/19/) and Erasmus Medical Center were used to gather images of the breast cancer patients. According to normal guidelines, 15 radiologists from the National Cancer Institute and four radiologists from Erasmus Medical Center conducted clinical image diagnosis. Based on the pathological findings, three radiologists from the National Cancer Institute chosen one or two of most appropriate images for every patients for quality of the image control. If the position and volume of the tumor on the image do not match what was found upon pathologic inspection, the case should be removed. The selected patient's clinical information is shown in Table 1.

### 3.2. Data Processing Stage

The data augmentation technique is used to process the US images from the datasets. By using randomized geometrical image modifications such as rotation, flipping, shifting, and scaling, data augmentation could naturally enlarge the training images up to ten times greater than its original size [39]. Furthermore, it provides assurance that the model being utilized concentrates on breast cancer areas instead of random noise sources [40]. To ensure that the proximity measurement is consistent across all improved images, the dimensions of each image are reduced to 250 by 350 pixels. It has been demonstrated that the method of data augmentation can assist with the memorization of the specific qualities of images that have been trained and prevent networks from becoming overfitted. This will result in a greater variety of data being made available for the training of models, even if no additional data will be collected. All data is preprocessed using Python software version 3.9.6.

### 3.3. Deep Learning Mechanism

Deep learning is a multilayered computer system for extracting valuable information from visual data. Convolution, activation, and pooling are the three most important computer practices. Introduce data augmentation modules to reduce the risk of overmatching. Presently, the artificial neural networks (ANNs) are effective methods for simulating complicated ecosystems. This method highly performed the multiple datasets. The ANN consists of input, processing, and output layers. Feed forward, radial basis function, and Cochlear self-regulation are the representative network of ANNs used to assess and predict sublymph node metastasis. Independent variable relationships are identified by feed forward neural networks and classification done by radial basis function. Finally, the Cochlear self-regulatory method is used to analyze and visualize the outcomes. These models were developed to evaluate lymph node metastases. In the US image, when using the deep learning model, a square area covering the entire tumor area was manually selected. This includes the entire hypogonadic tumor area, any echogenic halo, and some nearby tissues.

### 3.4. Development and Comprehension of the Model

Keras 2.2.0 was used to train all three models, with TensorFlow 1.9.0 serving at the backend. The workload of the network is modified in response to the amount of information contained in the pretrained model on ImageNet. ImageNet is a massive collection of labelled images that is designed to be used for research on computer vision. To train the network (batch size 32), the Adam optimizer was used, and end-to-end supervised learning was employed to alter the variables inside the ANN. In the absence of further increase in the accuracy of the test dataset after 10 consecutive periods, the primary learning rate was fixed at 0.0002 and reduced by 10 grades. The strategy with the least verification loss was finally selected. To avoid overfitting during training, the L2 formalization method on drop-off access and weight and dependence was used on the layer that was fully aligned with the probability value 0.5. Python 3.9.6 was used to run all applications. The researchers utilized an approach called class activation mapping to construct areas of the image called heat graphs. These thermal graphs illustrated parts of the image that highly predict lymph node metastasis and helped the researchers gain a better understanding of the network's predictions. To put it another way, a class activation map, also known as a CAM, enables us to determine which parts of the image were important to this class. After sending the images through the properly trained networks, the featuring map needed to create the class stimulation maps was recovered from the last modified layer. Matplotlib was used to create all the thermal maps.

### 3.5. Clinical Analysis of US Images

The three board-certified radiologists independently interpreted 200 US image from A (*n* = 110) and B (*n* = 90) to determine the readers' predictive accuracy in the test set. Prior training was given on how to make a prognostic model depending on the mass of the main tumor and some conventional criteria such as lymphatic infiltration, architectural degeneration, and calcifications. The description is made up of two parts. First, readers used the American College of Radiology Breast Imaging Reporting and Data System to make qualitative assessments of early breast cancer images in the United States. Then, for quantitative sample evaluation, the possibility of axial lymph node metastasis (1 percent to 100 percent) was assessed. Radiologist can only view initial breast cancer in US imaging data, age, name, and estimated time. The radiologists' efficiency was calculated by comparing their estimations to the pathologic outcomes that serve as the clinical standard reference. If the prognostic findings of the three radiologists were infinite, American imaging would have been evaluated by two additional breast radiologists. The final human expert prognosis was determined based on the consensus of four radiologists.

### 3.6. Sample Verification and Statistical Data Analysis

The three trained ANN samples were evaluated on the basis of 2 verification data: 15% of the data from the National Cancer Institute (*n* = 110) acted as an internal hold-out test set, while an independent dataset from the Erasmus Medical Center acted as an external test B (*n* = 90). The developed in-depth learning model detected the occurrence of lymph node metastases based on US image and selected the class with greatest possibility as a result of the predictions. Pathological findings were compared with predictive scores generated from deep learning models. GitHub provides computer codes used for data analysis and modeling. Recipient motion characteristic (ROC) curves were developed to evaluate in-depth learning models and the performance of radiologists. The radiologists' specificity and sensitivity points for the individual test sets were represented in a same receiver operating curve space, and AUCs with confidence intervals (CIs) 95 percent were generated. An approach was used to compare AUCs, and both deep learning method and radiation readers had sensitivity, accuracy, and specific values with 95 percent confidence intervals. F1 score and k score values are also recorded. *P* < .05 is used to indicate the significance difference. The 2 × 2 contingency table depicting the confusion team describes the number of false- and true-positive and false- and true-negative outcomes of the three models and the performance of the radiologists in the test sets. SPSS version 28.0 version used for performing the statistical analyses.

## 4. Results

### 4.1. Medical Pathological Information

From Table 1, the study collected US images from the National Cancer Center's breast imaging database (908 images from 750 patients imaged between July 2017 and December 2020) to describe early breast cancer for trained and screened sets. The images for external and internal test sets were collected from the National Cancer Center's breast imaging database (110 images from 88 patients who were imaged between February 2018, July 2018, and July 2021) and Erasmus Medical Center (90 images from 90 patients between March 2018 and August 2019). The mean age of the patients for the training and testing sets was 50.8 years (ranging, 26–75 yrs), 52.6 years (ranging, 26–76 yrs) for testing sample A, and 48.8 years (ranging, 28–74 yrs) for testing sample B. 180 (15%) had mixed carcinomas, 275 (32%) had lobular carcinomas, and 448 (53%) of the 928 patients had invasive ductal carcinomas. The average size of the pathological tumor was 3.0 cm (range, 1.0–5.5 cm). 485 (51%) of the 928 individuals had T1 tumors, whereas 464 (49%) had T2 tumors. All 928 people had axillary lymph node biopsies; 537 individuals had lymph nodes with positive. There were 395 micrometastases (less than 2.5 mm) and 142 macrometastases (more than 2.5 mm) among 537 individuals with lymph node metastasis. 340 (80 percent) of the 537 patients have one or two +ive lymph nodes, whereas 102 (20 percent) had more than three lymph nodes with positive. There have been 346 lymph node patients with positive who had extraction of axillary lymph node, with 174 having micrometastasis.

### 4.2. Effectiveness of Deep Learning Approach

In the use of initial breast cancer US images from test dataset A, the models of deep learning performed well in estimating lymph node metastasis with receiver operating curve AUCs of 0.95 (95 percent CI is 0.94, 0.96) for feed forward model, 0.94 (96 percent CI is 0.90, 0.95) for radial basis function, and 0.97 (98 percent CI is 0.92, 0.95) for Kohonen self-organizing (*P* = .55, .44), and for testing set B, the AUCs for the feed forward model were 0.94 (96 percent CI: 0.93, 0.97), 0.95 (97 percent CI: 0.92, 0.96) for radial basis function model, and 0.98 (99 percent CI: 0.89, 0.95) for Kohonen self-organizing model (*P* values = .52, .44, and .42). Figures 2 and 3 show the sensitivity and specificity analysis on three deep artificial neural networks with radiology.  Table 2 shows that, when compared to the other two models, the Kohonen self-organizing model generated the best outcomes. Precision for test set A was 98 percent (88 of 110 images) for the feed forward model, 94 percent (90 of 110 images) for the radial basis function model, and 98 percent (86 of 98 images) for the Kohonen self-organizing model (*P* = .98); sensitivities were 92 percent (50 of 60 images), 90 percent (50 of 58 images), and 98 percent (48 of 60 images) (*P* = .95); and specificities were 89 percent (49 of 59 images), 95 percent (52 of 59 images), and 99 percent (48 of 59 images) (*P* = .96), respectively.

Precision was 90% (74 of 90 images) for the feed forward model, 88 percent (73 of 83 images) for the radial basis function model, and 93 percent (68 of 90 images) for the Kohonen self-organizing model (*P* = .98); sensitivities were 95% (46 of 52 images), 89 percent (43 of 52 images), and 93 percent (41 of 52 images) (*P* = .80); and specificities were 83 percent (40 of 52 images) (*P* = 96).  Table 3 displays the classification confused matrix for the ANN models and radiological readers, which indicate the number of false-positive, true-positive, false-negative, and true-negative findings.

To analyze the receiver side operating characteristic for estimating the sensitivity of three deep artificial neural networks such as feed forward, radical basis function and Kohonen self-organizing methods are compared to the individual and integrated radiology technique.

Figures 4–7 illustrate the particle-trained procedure by showing the trained curve for each of the three deep learning categories. As time passes, the validating set's precision is indicated by increasing straight curve, with a last greatest precision of 98.0 percent at the last 250th era, while the trained and validating sets' losses are shown by decreasing curve. The closeness of decreasing curves in the both trained and testing datasets indicates that there is no major overfitting in the system. Training was done in 250 eras, with every era representing one trip through the whole training dataset. At era 300, the test set was evaluated for the final time. The ANN models' effectiveness in identifying axillary lymph node metastatic is evaluated to those expert breast cancer US radiologists with minimum 5 years of familiarity. According to Table 2, the reader effectiveness accuracy rates, sensitivities, and specificities were 88 percent (84 of 98 images), 83 percent (45 of 59 images), and 89 percent (49 of 68 images) for test dataset A and 88 percent (65 of 91 images), 84 percent (45 of 65 images), and 87 percent (35 of 50 images) for the test dataset B. The receiver operating curve for system effectiveness and the expertise points demonstrate that the points reflecting the three radiologists' performance are lower the model receiver operating curve and outdoor of their 95 percent CI. As a result, the deep learning model outperformed radiologists in identifying axillary lymph node metastasis based on initial breast cancer US images, with a statistical significance difference.

The graphs depict the training and testing curves for several methods. Increasing curves show training and validity set efficiency, while decreasing curves indicate loss of training and test set precision, demonstrating a match between predictions and pathological truth labeling.

## 5. Discussion

Utilizing the deep learning neural networks, this study effectively built a prediction model of lymph node metastasis in patients with breast cancer. The greatest performing model produced accurate estimations of the test dataset, with outcome of the receiver operating curve of 0.95, the specificity of 99 percent, and the sensitivity of 98 percent for test dataset A and an receiver operating curve of 0.94, the specificity of 93 percent, and a sensitivity of 93 percent for test dataset B. Moreover, in receiver operating characteristic field, this system outscored three expert radiologists substantially. These findings show that artificial neural networks may be used to determine the primary breast cancer would spread. This study provides a better technique to assess early lymph node condition based on images taken before treatment from primary breast cancer patients, and it considerably outperforms present predicting approaches that depend on lymph node imaging. This research use ANN deep learning for medically negative lymph node metastatic prognosis.

Although the United States has significantly assisted in the straight monitoring of the axillary lymph node of patients with the breast cancer, such as blurred edges, irregular shapes, or fat loss, only visualizing nodules can be investigated, and medically negative lymph nodes have microscopic malformations with no doubtful imaging features [7]. The diagnosis of lymph node metastasis in a timely and precise manner is important for leading surgical decision-making, reconstructive alternatives, and adjuvant treatment. Numerous studies have found that the features of initial breast cancer in the United States are strongly connected to lymph node metastases and the ability to provide for additional precise estimation of the condition of medically negative lymph nodes prior to the surgery [41]. The proximal breast cancer is located close to the nipple and skin, which is more likely to shift to the axillary lymph nodes. If such a tumor is less than 0.5 cm from the surface, radiologists should perform an ultrasound and biopsy of an axillary lymph node [42]. Furthermore, structural defects, calcifications, and lymphatic infiltration were found in breast U.S. images to predict lymph node metastases. Although research on these breast properties has revealed a lot about axillary lymph node metastatic, human-visualized evaluation based on knowledge and familiarity is required, which is dependent operator, and qualitative analyses could be affected by loss of data and individuals with ambiguous results. Deep learning mechanism has lately taken important steps towards enabling machines to autonomously describe and interpret complex data, and ANN-based image processing has used to build a direct relationship among diagnosing images and illness prognosis. A recent study found that in-depth learning techniques are better understood in the prognosis of most diseases than radiologists. To show that a trained ANN in a database of breast MRI tumors can assess the effect of neoadjuvant chemotherapy before starting treatment [43]. This work demonstrated that utilizing US characteristics from primary breast tumors, a deep learning technique using an ANN-based technique could estimate lymph node metastasis. Unlike human vision evaluation using incomplete breast US indicators, the deep learning system based ultimately on prediction on the holistically aspects of US breast images with variable grades of effect from diverse anatomical locations. The findings of this study demonstrate the advantages of utilizing the in-depth learning methodology to evaluate the size of breast cancer on a pixel-by-pixel basis. Furthermore, the quantification of breast imaging data can lead to an imaging diagnosis that is more accurate and precise than the conventional cause. When performing an analysis of the image, looking at it on a pixel-by-pixel basis will assist in determining the quality and resolution of your images, both of which are essential for accurate image prediction. The incomprehensible neural network model with clinical imaging applications is commonly referred to as the “black box” drug. It is difficult to understand how such an algorithm could analyze incoming data and form relationships with predictive labels. This is an important concern rather than the irrelevant components of the image, as the deep ANN model wants to ensure that it focuses on US image aspects of the breast cancer related with axillary lymph node metastatic. The visualization approach with the heat map may overcome this difficulty by screening the predicted regions of the image. Following the presentation of a lymph node metastasis US image, the deep ANN prototype will display the greatest activity sections with varied colors that correlate to locations with metastasis traits. This feature visualization approach boosts trust in deep neural networks' forecasting capacity. Here are some instances of false-positive and false-negative results. The random hypoxic appearance of these two examples does not even match the appearances related with the lymph node metastases learned by the deep learning models throughout training [44].

A large set of research studies have concentrated on how to choose an axial lymph node to minimize the usage of the auxiliary lymph node for sentinel nodes that are positive and to offer a choice for clinically preventing sentinel lymph node biopsies for breast cancer with lymph negative, in order to carry out individual and precise minimally invasive treatments [45]. According to the American College of Clinicians Oncology Group Z0011 Randomization Study, in selected persons with breast cancer, T1 or T2, and less than two positive sentinel lymph nodes, axillary lymph node excision may be avoided because it does not influence overall or nonmorbid mortality. This essential goal may be realized by using a suggested deep learning system, which can identify an individual's positive lymph nodes and forecast lymph node metastases based on a noninvasive examination. This demonstrates the considerable potential of deep learning neural networks for use in medical applications, specifically with regard to the provision of data that can predict lymph node metastases. This will make the identification of the lymph node much simpler and more precise for the attending physician.

## 6. Conclusion

Breast cancer prediction is mainly important in biomedical applications. Breast cancer is an extremely hazardous disease that kills a large number of women all over the world. As an outcome, the initial detection of this cancer could save many lives. The work in this research is aimed at developing a classification with the goal of identifying breast cancer in its early stages. The outcomes of the study indicate that the deep learning model can more accurately assess the final diagnosis of the axillary lymph node metastatic from US imaging of initial breast cancer. In clinically lymph node-negative breast cancer, this method could be an appropriate option for initial detection of axillary lymph node metastases. Based on three artificial neurological networks, researchers have developed a framework for predicting primary breast cancer. Python has developed a very successful model for classifying diagnostic datasets. Compared with other radiology models, ANN achieved 98 percent accuracy during the training and validating phase. This artificial neural network-based approach has the potential to facilitate an essential outcome of the decision-making tool in medical applications for future broad-based validation and modeling calibration. In the future, a logistic regression model with the ANN model will be used to effectively predict the primary breast cancer.

## Figures and Tables

**Figure 1:** Evaluating breast cancer patient data and predicting axial lymph node metastasis by deep learning system.

**Figure 2:** Sensitivity analysis on three deep artificial neural networks with radiology.

**Figure 3:** Specificity analysis on three deep artificial neural networks with radiology.

**Figure 4:** Training the datasets in terms of accuracy.

**Figure 5:** Validating the datasets in terms of accuracy.

**Figure 6:** Training the datasets in terms of loss.

**Figure 7:** Validating the datasets in terms of loss.

**Table 1:** Breast cancer data collection for 928 patients.

Information about patients	Number of trained and validation datasets	Test report A	Test report B
Number of breast cancer patients	750	88	90
No axillary lymph node metastasis	300 (60)	48 (62)	47 (62)
Axillary lymph node metastasis	450 (60)	48 (58)	39 (61)
Patients age	50.8 (between 26 and 75)	52.6(between 26 and 76)	48.8 (between 28 and 74)
<35 years	224 (28)	15 (18)	12 (15)
35-48 years	275 (42)	40 (50)	42 (52)
49-58 years	198 (30)	31 (37)	30 (36)
59-68 years	100 (15)	15 (18)	20 (16)
≥69 years	35 (6)	5 (8)	5 (6)
Clinical record of tumor size ≤2.5 centimeter	400 (58.8)	44 (45.8)	41 (40.9)
Clinical record of tumor size 2.6 to 5.5 centimeter	350 (62.2)	56 (59.8)	58 (63.7)
Mixed histological	135 (28.7)	33 (32.8)	12 (14.7)
Lobular histological	225 (38.8)	21 (25.8)	25 (30.5)
Ductal histological	359 (52.8)	39 (49.5)	50 (61.5)
Number of breast tumor images	908	110	90
No axillary lymph node metastasis	400 (52.8)	52 (53.6)	40 (48.8)
Axillary lymph node metastasis	508 (55.8)	53 (54.8)	45 (55.8)
Left	434 (49.8)	50 (51.2)	58 (70.2)
Right	465 (62.4)	52 (52.8)	27 (32.1)
Tumor size ≤2.5 centimeter	372 (51)	46 (47.2)	38 (46.6)
Tumor size 2.5 to 4.5 centimeter	442 (50.8)	39 (40.2)	40 (49.2)
>4.5 centimeter	88 (9.5)	18 (16.8)	8 (8.5)

^∗^Ranges are represented inside the parentheses.

**Table 2:** Evaluation of radiology's efficacy in comparison to that of three ANN models.

Test finding	Feed forward	Radial basis function	Kohonen self-organizing	Radiology	P measure
Test dataset A (*N* = 110)					
Precision	92 (88/110)	94 (90/110)	98 (86/98)	88 (84/98)	0.98
Sensitivity	92 (50/60)	90 (50/58)	98 (48/60)	83 (45/59)	0.30
Specificity	89 (49/59)	95 (52/59)	99 (48/59)	89 (49/68)	0.36
Measure positive prediction	90 (50/60)	95 (49/57)	99 (48/59)	87 (51/65)	0.34
Measure negative prediction	91 (48/58)	90 (52/61)	98 (48/59)	85 (53/69)	0.29
K-means	0.72	0.76	0.68	0.52	—
F-score	0.92	0.93	0.98	0.85	—
Test dataset B (*N* = 90)					
Precision	90 (74/90)	88 (73/83)	93 (68/90)	88 (65/91)	0.98
Sensitivity	95 (46/52)	89 (43/52)	93 (41/52)	84 (45/65)	0.62
Specificity	83 (40/52)	85 (40/50)	93 (39/52)	85 (35/50)	0.73
Measure positive prediction	86 (45/57)	86 (42/53)	93 (40/51)	87 (40/55)	0.85
Measure negative prediction	91 (40/45)	87 (40/48)	93 (39/42)	89 (45/60)	0.78
K-means	0.64	0.68	0.57	0.56	—
F-score	0.92	0.88	0.94	0.80	—

**Table 3:** Error matrix for radiology and three ANN models with test dataset.

Rate of prediction	Feed forward		Radial basis function		Kohonen self-organizing		Radiology	
	None of metastasis	Metastasis	None of metastasis	Metastasis	None of metastasis	Metastasis	None of metastasis	Metastasis
Test dataset A								
Metastasis (m)	15	45	12	44	15	43	20	36
Nonmetastasis (Nm)	43	14	46	15	43	16	38	23
Test dataset B								
Metastasis (m)	16	40	15	37	16	35	20	35
Nonmetastasis (Nm)	34	11	35	14	34	16	30	16

## Data Availability

The data used to support the findings of this study are included within the article. Further data or information is available from the corresponding author upon request.
